# Olive Disease Classification Based on Vision Transformer and CNN Models

**DOI:** 10.1155/2022/3998193

**Published:** 2022-07-31

**Authors:** Hamoud Alshammari, Karim Gasmi, Ibtihel Ben Ltaifa, Moez Krichen, Lassaad Ben Ammar, Mahmood A. Mahmood

**Affiliations:** ^1^Department of Information Systems College of Computer and Information Sciences, Jouf University, Jouf, Saudi Arabia; ^2^Department of Computer Science, College of Arts and Sciences at Tabarjal, Jouf University, Jouf, Saudi Arabia; ^3^ReDCAD Laboratory, University of Sfax, Sfax, Tunisia; ^4^STIH, Sorbonne University, Paris, France; ^5^Faculty of CSIT, Al-Baha University, Al Bahah, Saudi Arabia; ^6^College of Sciences and Humanities, Prince Sattam Bin Abdulaziz University, Al-Kharj, Saudi Arabia; ^7^Department of Information Systems and Technology, FGSSR, Cairo University, Egypt

## Abstract

It has been noted that disease detection approaches based on deep learning are becoming increasingly important in artificial intelligence-based research in the field of agriculture. Studies conducted in this area are not at the level that is desirable due to the diversity of plant species and the regional characteristics of many of these species. Although numerous researchers have studied diseases on plant leaves, it is undeniable that timely diagnosis of diseases on olive leaves remains a difficult task. It is estimated that people have been cultivating olive trees for 6000 years, making it one of the most useful and profitable fruit trees in history. Symptoms that appear on infected leaves can vary from one plant to another or even between individual leaves on the same plant. Because olive groves are susceptible to a variety of pathogens, including bacterial blight, olive knot, *Aculus olearius*, and olive peacock spot, it has been difficult to develop an effective olive disease detection algorithm. For this reason, we developed a unique deep ensemble learning strategy that combines the convolutional neural network model with vision transformer model. The goal of this method is to detect and classify diseases that can affect olive leaves. In addition, binary and multiclassification systems based on deep convolutional models were used to categorize olive leaf disease. The results are encouraging and show how effectively CNN and vision transformer models can be used together. Our model outperformed the other models with an accuracy of about 96% for multiclass classification and 97% for binary classification, as shown by the experimental results reported in this study.

## 1. Introduction

If there is one field that is currently in full development, it is that of artificial intelligence [1, 2]. From disease classification and segmentation [3, 4] to facial recognition to conversational assistants, autonomous vehicles, and online shopping recommendation systems, these new technologies are invading our daily lives. And in this broad field, one type of method in particular is the talk of the town: but between the potential and what we should really expect from it, between deep learning and other areas of artificial intelligence [5, 6], it is not necessarily easy to navigate. So the researchers wanted to take a closer look at this topic, particularly to figure out where we are in the field of agriculture. In fact, deep learning in agriculture [7] has been explored for some time, first in research and then in RD. At a time when the first commercial applications will be coming to market, it seems important to us to take an enlightened look at these technologies: to understand what they are, what applications there are, what their limitations are, and what questions are still open.

Agriculture and plants play an important role in boosting a country's economy. Diseases in the leaves of many plants such as fruits, olive trees, citrus fruits, rice, guava, and wheat can have a significant impact on their productivity. Therefore, it is critical to protect crops from infections at an early stage so they can be treated quickly. Early detection and prediction of plant diseases is one of the most important prerequisites for improving agricultural cultivation.

Olive tree is attacked by many types of pathogens such as bacteria. Before reaching maturity, the diseases in the leaves of the olive tree can have a significant impact on its production. Therefore, rapid and accurate diagnosis of leaf diseases is necessary, as early as possible. Human intervention-based leaf disease detection is needed to address this problem.

The adoption has been led by recent advances in computer vision and artificial intelligence. Deep learning techniques [8, 9] have been widely applied in computer vision task especially image classification. In this paper, we address the problem of diseases on olive leaves. In particular, we propose a hybrid deep learning based model for olive disease classification. To prove our approach, we use a dataset that was obtained over the spring and summer that was used by us in the process of evaluating our proposed ideal model that is based on deep learning. This dataset includes 3,400 olive leaves that were separated into three distinct categories: healthy leaves, leaves infected with *Aculus olearius*, and leaves infected with olive peacock spot.

The main contributions of this paper are as follows:

1. To improve the quality of olive images, we use the median noise filtering algorithm that removes and reduces noise after data augmentation process.
2. We propose a hybrid deep learning-based architecture that combines the convolutional neural network (CNN) model and the vision transformer model to extract the most relevant features from olive images.
3. For the image classification process, we use a pooling layer and dropout to avoid the overfitting problem before applying a softmax feature.

The rest of this paper is organised as follows: In Section 2, we review recent relevant work on olive disease diagnosis and classification.  Section 3 presents the proposed olive oil disease classification model.  Section 4 describes the experimental evaluation of our model and discusses the results with corresponding analyses. Conclusions and future work are discussed in Section 5.

## 2. Related Work

Several works have been proposed for the diagnosis of diseases affecting plant leaves, especially olive leaves [10]. These works focused on the analysis, detection, and classification of many plant diseases using numerous image processing and deep learning techniques [11, 12].

Several approaches have been proposed for diseases detection using different deep learning techniques [13–15]. Authors in [13] developed a model that can detect plant diseases by smartphones applications. In [16], the authors addressed the problem of early detection of anthracnose in olives. The study conducted is based on the application of advanced deep learning techniques and CNN architectures to hyperspectral images. The dataset includes hyperspectral images in the visible (VIS) and near infrared (NIR) regions. Moreover, authors in [17] proposed a hybrid model that uses deep learning techniques for sunflower diseases recognition and classification. In particular, they used two deep learning models: VGG-16 and MobileNet, for classification purposes. In [18], the authors propose a new image analysis technique for olive disease detection and classification. These techniques are based on image texture features detected on the olive plant leaf. The first analysis technique uses histogram thresholding and k-means segmentation to isolate the infected area. The second analysis technique uses first- to fourth-order moments to detect the relationship between the infection and one or more texture features.

Deep learning-based approaches have found wide application in the field of plant disease identification and classification [19, 20]. CNN is an efficient model that aims to extract autonomous features. It has proven to be very efficient in detection and classification tasks due to its powerful deep learning structure: self-learning, adaptability, and generalization [21]. However, CNN require a large amount of training data and a set of parameters to be fixed. Several works have addressed the requirements of CNN [22, 23]. The authors in [24] provided an overview of the importance of deep learning as a current research focus in agricultural crop protection. In particular, the authors analyzed existing work on leaf disease detection based on image processing, hyperspectral imaging, and deep learning techniques. The review of the literature clearly showed that most of the works provided evidence that deep learning techniques are the best tool for leaf disease detection. Therefore, collecting a large amount of data has a great impact on obtaining highly accurate results. The datasets used are manipulated by data augmentation techniques, transfer learning techniques, and the use of a CNN. Although the results of previous work are sufficient, the problem of plant disease detection still needs to be addressed, as the lack of labels on the data can affect the quality of pixels representing disease symptoms. Moreover, in [22], the authors proposed a study of olive leaf disease classification using transfer learning techniques on deep CNN architectures. A set of 3400 images of healthy leaves was used to validate the working method. The experiments were performed with and without data augmentation. The obtained results clearly show the importance of data augmentation. After these experiments, the Adam and SGD optimization algorithms were applied to obtain more accurate results. The authors in [25] have proposed a deep CNN-based model for olive disease detection and classification. The proposed model uses a parameterized transfer learning model with data augmentation and probably outperforms other methods in terms of accuracy and precision, but it takes a lot of time to train. A deep learning architecture is applied in [26] to classify several leaf diseases of plants and fruits. In summary, a deep transfer learning model was used to learn features. Several support vector machine models are used with the radial basis function to improve feature discrimination. The results showed the potential of the proposed hybrid model based on the modified deep transfer learning network and the set of learning models for leaf disease classification.

## 3. Proposed Model for Olive Disease Classification

In this section, we will discuss the hybrid deep learning model we proposed for olive disease classification.  Figure 1 provides a summary of this methodology for our consideration. The architecture of the approach can be divided into three steps. In the first step of the method, preprocessing of the dataset is performed to remove noise and improve image quality. This is done using an algorithm known as a noise filter. After that, a data enhancement procedure is performed. The preprocessed dataset is then fitted with the hybrid model previously described, which is composed of CNN models and vision transformers, to extract features from it. It is important to note that the primary goal of using such a variety of models is to run a series of experiments to determine which results are most favorable. The third and final step is image classification using a pooling layer and dropout to avoid the problem of overfitting before applying a softmax function. This stage is used before the last stage.

### 3.1. Data Augmentation

At this stage of the process, the median noise filtering [27] method is applied to the images to enhance them. The median filter is a more effective means of removing or reducing noise in the collected photographs because it replaces a pixel with the median of the gray levels that are in the immediate vicinity of the pixel [28]. Research has demonstrated that data augmentation can be used effectively in image categorization [29].

There are studies that compare basic techniques such as cropping, rotating, and spinning images with more advanced techniques such as Generative Adversarial Networks (GANs) for generating images of different styles or neural network augmentation approaches to learn which augmentations improve a classifier the most. Cropping an image, rotating an image, and flinging an image are all examples of basic techniques. Despite the proposed models, text augmentation methods have not been studied nearly as thoroughly as image augmentation methods.

Altering the photos in a data collection can include geometric changes such as rotating, shifting, scaling, or flipping the images. Data augmentation not only improves the generalizability of models or models that prevent overfitting, but also improves results in unbalanced classification tasks. In other words, models that prevent overfitting are improved by data augmentation.

### 3.2. Hybrid Feature Extraction Method

Convolutional neural networks have contributed significantly to deep learning achievements in visual tasks in recent years [30, 31]. This is in part due to the strong inductive bias of spatial equivariance encoded by convolutional layers, which have been shown to be essential in learning general purpose visual representations for ease of transfer and high performance. Remarkably, however, recent research has shown that neural transformer networks perform equivalently or even better in classifying images when applied to large datasets. The operation of these vision transformers (ViT) is almost identical to that of transformers used in speech citations devlin2018bert. Instead of convolution, these vision transformers (ViT) use self-awareness to aggregate information across different locations. In contrast, much past work has focused on explicitly adding image-specific inductive biases [32, 33].

Image classification networks based on CNN tend to transmit representations with a decreasing level of resolution. ResNet, for example, consists of five stages, with each stage decreasing the resolution by half, resulting in a final feature map that is 1/32*∗*1/32 in each dimension. In ViT, on the other hand, tokens are initially set to a size of 16 × 16, which reduces the resolution in that dimension; yet the final layer continues at that resolution. As a result, ViT is more likely to retain location information than ResNet. It is not possible to say that ViT has an advantage over ResNet because it retains location information, since image classification tasks do not require location information for classification decisions.

In addition, the strategy of gradually reducing resolution, similar to ResNet, has been widely used in recent studies of vision transformers. An example of this is the pyramid vision transformer, shown in the figure above on the right. Transformer systems use self-awareness, and the memory required to store an image grows proportionally with the fourth power of its size. This makes it difficult to process large resolutions, but by using a strategy that gradually reduces resolution, as is the case with CNN systems, it is possible to process high-resolution information in the first layer while saving storage space. This is achieved by a technique similar to that used in CNN systems.

### 3.3. AlexNet

Researchers use AlexNet as one of the deep learning models. AlexNet's network architecture consists of a total of eight layers. The first five layers are convolutional layers, while the last three layers are fully connected layers. It improves the training performance of the activation function by using the tanh and sigmoid functions as described in [30]. An illustration of the AlexNet model can be seen in Figure 2.

### 3.4. VGG

The acronym VGG stands for Visual Geometry Group, and its architecture is a conventional deep convolutional neural network (CNN) with multiple layers. When we refer to the VGG-16 or VGG-19 models, “deep” refers to the number of convolutional layers, which is 16 and 19, respectively.

Innovative new models for object recognition can all be traced back to the VGG architecture as a model. VGGNet, designed as a deep neural network, outperforms the baseline performance of many other tasks and datasets in addition to ImageNet. Moreover, it is currently considered one of the most widely used designs for image recognition.

The VGG19 model, sometimes referred to as VGGNet-19, is conceptually identical to the VGG16 model except that it supports 19 layers. The numbers “16” and “19” refer to the total number of weighting layers (convolutional layers) included in the model. This shows that VGG19 is more advanced than VGG16 in terms of the number of convolutional layers.

The VGG network is constructed using extremely small convolutional filters as building blocks. Thirteen convolutional layers and three fully connected layers make up the VGG-16. Let us first take a brief look at the architecture of the VGG platform: Input: the VGGNet accepts images with a size of 224 × 224 pixels as input. For the ImageNet contest, the developers of the model removed the 224 × 224 pixel area from the center of each image. This ensured that the input size of the image remained the same. Convolution layers: The convolutional layers of the VGG use a minimum receptive field denoted by the notation 3 × 3, which is the smallest size still capable of capturing left/right and top/bottom information. In addition, there are 1 × 1 convolution filters that perform the function of a linear transformation on the input. This is followed by a ReLU unit, a significant innovation from AlexNet that reduces the time required for training. The acronym “ReLU” stands for “rectified linear unit activation function.” This type of piecewise linear function outputs the input when it is positive but returns zero when the input is negative. To maintain the same spatial resolution after convolution, the convolution step was set to a constant value of 1 pixel (step is the number of pixel shifts over the input matrix). Hidden layers: The entirety of the hidden layers of the VGG network is driven by ReLU. Local Response Normalization (LRN) is generally not used by VGG because it increases memory requirements and the time needed for training. It also does not noticeably improve overall accuracy. Fully linked layers: The VGGNet consists of three fully linked layers. In the first two of the three levels each has a total of 4096 channels, while the third level has only 1000 channels, with one channel associated with each class.

The difference: although it is based on AlexNet, VGG has some special features that distinguish it from other competing models, including the following.

VGG uses very small receptive fields, unlike the massive receptive fields used by AlexNet (11 × 11 with a stride of 4), (3 × 3 with a stride of 1). The decision function is much more discriminative than before, as there are now a total of three ReLU units instead of just one. There are also fewer parameters (27 times the number of channels as opposed to 49 times the number of channels in AlexNet). The decision function in VGG becomes more nonlinear due to the inclusion of 1 × 1 convolutional layers, with no impact on the receptive fields. Due to the modest size of the convolution filters, VGG is able to use a large number of weighting layers. As might be expected, the larger number of layers results in better overall performance. However, this is not a particularly unusual property.

### 3.5. Vision Transformer (ViT) Model

The transformer architecture developed by the authors in [34] is currently at the forefront of innovation in the field of natural language processing (NLP). Dosovitskiy came up with the idea for the vision transformer (ViT) architecture for image classification application after observing the effectiveness of the self-attention-based deep neural networks of transformer models in natural language processing (NLP). The general training procedure for these models is based on decomposing the input image into individual fields and then treating each embedded field as if it was a word in a natural language processing system. These models use self-observation modules to discover the connection between the embedded patches. Because of the exceptional performance of ViTs, numerous researchers have investigated ViT models for a variety of vision tasks [35]. In the area of object recognition, Carion et al. [33] proposed a new architecture for object recognition systems using an asset-based global loss and a transformer-encoder-decoder algorithm. They showed results equivalent to the dominant R-CNN method on the challenging dataset COCO.

The established architecture proposed by Steiner corresponds to the original ViT design presented by Dovosviky, except that the MLP header was replaced by a linear classifier.  Figure 3 gives an overview of the ViT design architecture that you can view. In summary, a ViT model starts with segmenting the input image into different subimages. The transformer encoder receives a sequence of 1D patch embeddings as input and then uses self-observation modules to compute the relationship-based weighted sum of the outputs of each hidden layer. This is done by feeding the sequence into the encoder. Thanks to this technique, the transformers are able to understand the global dependencies contained in the input images.

### 3.6. Classification

The structure of multilayer neural networks consists of three layers: an input layer, one or more hidden layers that are sequentially switched from the input layer, and an output layer. The first layer of multilayer neural networks is always connected to the outside of the network or to more than one outside of the network.

At this stage of the process, our attention was focused on the last layer to obtain the best answer. To this end, we combined the features identified in the previous phase and used them as input to our classifier, which is based on a softmax layer. In this way, we were able to determine which answer was the most accurate.

Compared to the activation function of the hidden layers, the activation function of the output layer is unique. The function of each layer is different, as is the way it is implemented. When a classification task is completed, the last layer allows creating class probabilities for the input data.

(1) $$\begin{array}{c} \text{Soft}\max\left(x_{i}\right)=\frac{\exp\left(x_{i}\right)}{\sum_{j}\exp\left(x_{j}\right)}. \end{array}$$

It is a vector in which each of the elements, denoted by *x*_*i*_, is a value and it can have any value in the real world. Since the sum of the output values of the function must equal 1, the lowest term is the normalization term, which ensures that the probability distribution is valid. This condition must be satisfied for all output values of the function.

Because they are capable of training enormous amounts of data with a large number of parameters in an efficient and accurate manner, deep neural networks are the learning methods that have received the most attention in published papers. Nevertheless, overfitting is one of the challenges faced by these types of networks. One of the several strategies available to combat the problem of overfitting is called regularization and involves the use of the dropout function. The use of the dropout function has the advantage of allowing the combination of different networks in a single architecture, while limiting overmatching between units. It is well known that the dropout function performs excellently in fully connected layers as well as in pooling layers.

## 4. Experiment Results and Discussion

This section discusses the results of the experimental tests conducted with the model described in this study.

Using our own adapted deep learning model, we also compare the results of different deep learning approaches. Python was used in the development of this model, and Google's deep learning server supported its deployment.

To test the applicability of our proposed model, we conducted a series of experiments with deep learning approaches. Our model considers two different approaches. The first one concerns the categorization task, where images are divided into two classes (binary classification). The second one is about the transition from a binary classification system to a multiclass system. Our dataset was classified into the following categories: “healthy,” “pea cock spot,” and “*Aculus olearius*.”

### 4.1. Dataset Description and Evaluation Metrics

A dataset that was obtained over the spring and summer was used by us in the process of evaluating our proposed ideal model that is based on deep learning. With the assistance of an agricultural engineer who is highly knowledgeable in the subject matter, 3,400 olive leaves were separated into three distinct categories: healthy leaves, leaves infected with *Aculus olearius*, and leaves infected with olive peacock spot. Our dataset also included uninfected olive leaves. We provide an illustration of a sample photo along with descriptions of the various olive diseases that can be found at Figure 4.

Table 1 shows that the data set was divided into two groups, 80 percent of which were used for training and 20 percent for testing. The results of the CNN model can be negatively affected by anomalies in the distribution of data sets when they are split into training and testing groups. In creating the training and test groups, we used k-fold cross-validation to avoid this problem.

To evaluate the performance of the proposed model as well as other deep learning methods, we used standard metrics used in large image sets to estimate classification tasks, such as accuracy and precision, recall, and *F*-measure.

Since this is an unbalanced problem and the accuracy measure is derived by predicting that all observations belong to the majority class, which leads to spurious results, we selected all of these measures. It was therefore imperative that the categorization process produces reliable results, so we included additional metrics:

(2) $$\begin{array}{c} \text{Accuracy}=\left(\frac{\left(\text{TP}+\text{TN}\right)}{\left(\text{TP}+\text{FP}+\text{TN}+\text{FN}\right)}\right),\\ \text{Precision}=\left(\frac{\text{TP}}{\left(\text{TP}+\text{FP}\right)}\right),\\ \text{Recall}=\left(\frac{\text{TP}}{\left(\text{TP}+\text{FN}\right)}\right),\\ F1-\text{score}=2*\left(\frac{\left(p*R\right)}{\left(P+R\right)}\right),\\ \text{TPR}=\left(\frac{\text{TP}}{\left(\text{TP}+\text{FN}\right)}\right),\\ \text{FPR}=\left(\frac{\text{FP}}{\left(\text{FP}+\text{TN}\right)}\right), \end{array}$$

where TP refers to true positives, FP refers to false positives, P refers to precision, R refers to recall, TPR refers to the rate of true positives, and FPR refers to the rate of false positives. We use the python package sklearn3 and the Keras application 4 for deep learning models in order to compare the results of many deep learning approaches that we investigate as part of our research. This is an important aspect of our work.

### 4.2. Evaluation of Deep Learning Model

In this section, we evaluate and compare the effectiveness of different deep learning models, including AlexNet, VGG-16, VGG-19, and Transformer ViT, to determine the most effective classifier for olive disease diagnosis. The aim of this study is to evaluate the effectiveness of different deep learning models in classifying olive diseases. The results of the binary and multiple classifications are shown in Table 2.

In the first scenario, the transformer and VGG-16 models obtained the best results in terms of average accuracy. These two models obtained values of 0.96 and 0.89, respectively. It is important to mention that the transformer classifier had the highest overall accuracy, calculated at 0.96, and it outperformed all other classification methods in terms of accuracy rate. This can be explained by the fact that transformer is a deep learning method for categorization. It works well when the variable to be predicted is binary, assuming that all predictors are independent of each other, and works under the assumption that there are no missing values in the data. Moreover, the VGG-19 classifier algorithm had a prediction accuracy of 0.84, which is the lowest overall accuracy. On the other hand, in the second case, it is observed that the result of transformer is always better when classifying into several groups, including “healthy,” “olive peacock spot,” and “*Aculus olearius*.” Therefore, the expected highest classification accuracy of the transformer classifier approach was 0.95. The results clearly showed that the transformer classifier performed much better than any other classification approach in both cases.

Consequently, the transformer classifier is an option worth considering for both binary and multiclass classification. Nevertheless, this result was not sufficient. We not only focus on deep learning methods, which are widely known to perform strongly in classification, but also incorporate other advanced hybrid deep learning methods for optimal classification. In this way, we aim to ensure that our evaluation is as applicable as possible for practitioners. With this in mind, we proposed that they change their basic architecture by adopting a hybrid strategy for the feature extraction process as a solution to this problem. We believe that this adaptation has the potential to significantly improve the overall quality of the results. We propose to use a hybrid deep learning model that combines the transformer and CNN models to achieve better results.

### 4.3. Evaluation of Hybrid Deep Learning Model

The results obtained by the hybrid deep learning models based on transformer and CNN models are presented in Table 3 for two different binary and multiclassification scenarios. In the first scenario, the results classifying our dataset into two categories are presented. In the second scenario, the results for the different types of diseases are presented. These include “healthy,” “olive peacock spot,” and “*Aculus olearius*.” We note that the best results for the binary classification were obtained by hybridising the ViT and VGG-16 models and that this model gave results close to 0.97.

The second section of Table 3 provides a summary of the outcomes that were obtained through the application of hybrid deep learning models that were based on a transformer model for multiclass categorization. It has come to our attention that this hybrid model was successful in achieving the best outcomes for multiclass classification, with the maximum accuracy of approximately 0.96.

The results of our experiments have shown that our proposed model, which is based on a hybrid approach, improved both our accuracy and our precision; nevertheless, the feature in which we saw the biggest improvement was significance.

In conclusion, the development of neural networks, which emerged as a branch of deep learning techniques, has made it possible to solve seemingly simple issues such as classifications in a significantly amount of time. In particular, it is extremely evident that our improved hybrid deep learning model for identifying olive leaf diseases has produced excellent results and has attained a high classification accuracy rate. This can be seen from the fact that the model has given satisfactory results. Because of this, we are able to point out that the model that we have proposed, which is based on a hybrid algorithm, makes an effort to categorize the dataset by locating an important feature for the presentation of the images and provides a high diagnostic of olive leaf images.

### 4.4. Evaluation of Optimized Hybrid Model for Binary and Multiclassification

To achieve the best possible prediction scores from the models that were developed was one of the overarching objectives of this study. When the models are constructed in accordance with their architectural frameworks, the values of specific parameters are essential to increasing the success rate of predictions. In the context of deep learning and machine learning, the term “loss” refers to the disparity between the values that were predicted and those that were actually observed; achieving the lowest possible loss indicates high model performance. In order to ensure that there are fewest possible losses, it is necessary to minimize the model's loss function. To solve this problem, optimization strategies like Adam [36], AdaGrad [37], and RMSProp [38] could be utilized. It is possible that the way each approach works to get the global minimum, also known as the value with the fewest losses, will be different. Investigating the effect that these methods have on the three models that were produced has consequently been one of the key focuses of this research. As a direct consequence of this, these four strategies have been evaluated for their potential to optimize networks.

According to Table 4, Adam achieved an accuracy of 0.97 for binary classification and 0.96 for multiclassification, while AdaGrad earned an accuracy of 0.86 and 0.89, respectively. The Adam optimization strategy was found to outperform the other two models in this study's tests.

## 5. Conclusion

In this research, we proposed a hybrid deep learning model for olive leaf disease classification. To achieve this, we used three different deep learning models in addition to a modified vision transformer model. The main objective of our proposed strategy was to identify the best possible feature and ensure higher accuracy. Before proceeding to the evaluation of the proposed strategy, we first evaluated the results of several different deep learning models. The models were trained and validated using a database containing 3,400 different images of olive leaves. Compared to other deep learning models, the results showed that the accuracy of the vision transformer model was the highest. We put our hybrid deep learning models to the test by using them to classify data into binary and multiclass categories.

Compared with other deep learning models, including VGG-16, VGG-19, and vision transformer, we found that the accuracy rate of the hybrid deep learning models was significantly higher than that of the other deep learning models. In binary classification, the most effective model, which was a combination of the ViT model and the VGG-16 model, achieved an accuracy rate of 97 percent. We intend to adapt the most effective deep learning model to other plant collections in the future, and we will strive to collect more photos of olive diseases.

## Figures and Tables

**Figure 1:** Proposed model for olive disease classification.

**Figure 2:** Architecture of AlexNet.

**Figure 3:** Vision transformer architecture.

**Figure 4:** Slices of typical images with three types of the olive diseases findings: (a) healthy; (b) *Aculus olearius*; (c) peacock spot.

**Table 1:** Dataset description.

Class name	Training set	Testing set	Total
Healthy	830	220	1,050
Olive peacock spot	1,200	260	1,460
*Aculus olearius*	690	200	890

**Table 2:** Evaluation of deep learning model for binary and multiclassification.

	Binary classification			
	Accuracy	Precision	Recall	fBeta
AlexNet	0.82	0.89	0.84	0.85
VGG-16	0.89	0.91	0.89	0.90
VGG-19	0.84	0.86	0.85	0.86
Transformer (ViT)	0.96	0.97	0.96	0.96

	*Multiclassification*			
AlexNet	0.84	0.86	0.87	0.86
VGG-16	0.85	0.87	0.86	0.87
VGG-19	0.82	0.75	0.94	0.84
Transformer (ViT)	**0.95**	**0.94**	**0.98**	**0.96**

**Table 3:** Evaluation of proposed model based on optimized algorithms for binary and multiclassification.

	Binary classification (ViT + VGG-16)			
	Accuracy	Precision	Recall	fBeta
ADAM	**0.97**	**0.98**	**0.98**	**0.98**
RMSProp	0.82	0.89	0.84	0.85
AdaGrad	0.86	0.91	0.87	0.89

	Multiclassification (ViT + VGG-16)			
ADAM	**0.96**	**0.97**	**0.96**	**0.96**
RMSProp	0.86	0.92	0.80	0.86
AdaGrad	0.89	0.91	0.87	0.89

**Table 4:** Evaluation of hybrid deep learning model.

	Binary classification			
	Accuracy	Precision	Recall	fBeta
ViT + VGG-16	**0.97**	**0.98**	**0.98**	**0.98**
ViT + VGG-19	0.96	0.98	0.96	0.97
Transformer (ViT)	0.96	0.97	0.96	0.96

	*Multiclassification*			
ViT + VGG-16	**0.96**	**0.97**	**0.96**	**0.96**
ViT + VGG-19	0.95	0.96	0.95	0.95
Transformer (ViT)	0.95	0.94	0.98	0.96

## Data Availability

The Olive dataset used to support the findings of this study has been deposited in the https://github.com/sinanuguz/CNN_olive_dataset. Comparing the outcomes of various deep learning methods is also part of our research and specially vision transformer model; for that, we use https://keras.io/examples/vision/image_classification_with_vision_transformer/ as a python package and Keras application (https://www.tensorflow.org/api_docs/python/tf/keras/applications) for deep learning models.
